# Radial Expansion Favors the Burrowing Behavior of *Urechis unicinctus*

**DOI:** 10.1155/2023/2478606

**Published:** 2023-10-04

**Authors:** Shanpeng Li, Yun Zhang, Ruihua Zhang, Jianlin Liu

**Affiliations:** ^1^College of Engineering, Lishui University, Lishui 323000, China; ^2^State Key Laboratory of Solid Lubrication, Lanzhou Institute of Chemical Physics, Chinese Academy of Sciences, Lanzhou, Gansu 730000, China; ^3^College of Pipeline and Civil Engineering, China University of Petroleum (East China), Qingdao 266580, China

## Abstract

*Urechis unicinctus* can utilize the ability of large deformation to advance in sands by radial expansion, just using a small force. However, the large deformation of *U. unicinctus* skin and the discrete nature of the sands make it hard to analyze this process quantitatively. In this study, we aim to uncover the burrowing mechanism of *U. unicinctus* in granular sediments by combining discrete and finite elements. We observe that *U. unicinctus* will expand radially at the head, and then the head will shrink to move forward. The radial expansion will collapse the sands and let them flow, making it easy to advance. *U. unicinctus* mainly relies on the skin's large deformation and sufficient pressure to achieve radial expansion. Thus, we first establish the large deformation constitutive model of the skin. The stress–strain relationship can be expressed by the Yeoh model. Meanwhile, the pressure required for radial expansion is indirectly measured by the balloon experiment. To study the effect of radial expansion on the burrowing behavior, we use the finite element method–discrete element method (FEM–DEM) coupling model to simulate the expansion process of burrowing. The simulated pressure for radial expansion is very close to the experimental data, verifying the reliability of the simulation. The results show that the expansion can drastically reduce the pressure of sand particles on the head front face by 97.1% ± 0.6%, significantly decreasing the difficulty of burrowing. This unique underwater burrow method of *U. unicinctus* can provide new ideas for engineering burrowing devices in soft soil, especially for granular sediments.

## 1. Introduction

When some engineering equipment, such as ship's anchor and cable laying equipment, advance in underwater sands, the resistance of the sands will gradually increase with the increase of the depth, making the objects challenging to travel [1]. It is of great technical significance to make the burrow in sands an easy thing. Driven by the survival pressure, animals have evolved many unique ways of burrowing in the mud or granular substrates, including undulatory locomotion, dual-anchor mechanism, and peristaltic motion. As for undulatory locomotion, the desert-dwelling sandfish (*Scincus*) can swim in sands and overcome resistance by propagating an undulatory traveling wave [2]. The ratio of the undulation amplitude to the wavelength determines the sand-swimming performance of sandfish in the subsurface [3]. Anguilliform fish (*Pisodonophis boro*) also uses lateral undulation to penetrate and move in sandy sediments underwater with a high slip factor [4]. More interestingly, nematodes (*Caenorhabditis elegans*) can locomote a greater distance through the fluctuations of swimming in the saturated soil than in the fluid without particles [5]. The second burrowing mechanism is a dual-anchor mechanism used by bivalves [6]. The clam (*Ensis directus*) burrows downward sands by the joint action of shell and foot movement and out of sands by simply extending and contracting its foot [7].

The peristaltic motion is another common burrowing way, inducing crack propagation in elastic muds. The earthworm *Lumbricus terrestris* burrows by forcefully enlarging cracks through the radial expansion in the soil [8]. Due to the huge energy consumption of excavation, some earthworms can reuse existing caves to build nests [9]. Inspired by its adapting to terrestrial environments, new geotechnical in situ testing devices are explored to simulate the adaptations of earthworms developed for soil penetration [10]. An earthworm-inspired robot is created for internal maintenance in long and thin pipelines employing its unique creeping mode [11]. Apart from earthworms in terrestrial environments, clam worms (*Nereis virens*) in marine sediments can utilize the repetitive expansion of the head to promote crack propagation and advance in muddy and cohesive sediments consuming very little energy [12]. More accurate forces for crack propagation are measured in gelatin by the photoelastic stress analysis based on sediment mechanics [13]. Similarly, the glycerid polychaete *Hemipodus simplex* can produce forces larger than that necessary to extend the crack by fracture, which will plastically deform the mud to build a semipermanent burrow [14]. However, the crack propagation induced by the peristaltic motion is not a viable penetration mechanism in granular substrates. Therefore, it is meaningful to explore the mechanism of creeping in the sand, which may reduce the difficulty of advancing in the sands for some construction machinery, such as the ship's anchor and cable laying equipment.

*Urechis unicinctus* (Echiura, Annelida), commonly known as sea intestine, can advance in sands by a unique peristaltic motion, i.e., huge radial expansion and shrink. *U. unicinctus* lives in U-shape burrows in the subtidal zone and has high nutritional and medicinal values, rapidly promoting its aquaculture [15, 16]. Existing studies mainly focus on its nutritional components, medical value, and environmental tolerance [17, 18]. However, there are few studies on *U. unicinctus* from the perspective of mechanics, which is the key to revealing the burrowing mechanisms in sands. Meanwhile, it should be noted that *U. unicinctus* can flexibly achieve shrinkage, expansion, and twisting [19] due to the large deformation of its skin. Although there have been many studies on the constitutive model of skin [20–25], it is not yet clear about the *U. unicinctus* skin's mechanical properties of large deformation. Thus, in the present study, we focus on the burrowing mechanisms of *U. unicinctus* in sands. Considering the vigorous development of bionic soft robots in the fields of crawling [26, 27], jumping [28, 29], swimming [30], walking [31, 32], and rolling [33], this exploration could be beneficial for manufacturing soft robotic creeping devices and machines [34].

## 2. Materials and Methods

### 2.1. Animal

To eliminate the influence of individual activity differences, some *U. unicinctus* bought from the seafood market are kept in a fish tank with 80×60×100 cm^3^ for 1 day, where seawater salinity is 1.024 and temperature is 20°C. We select active *U. unicinctus* with a uniform size for study to avoid the influence of the body size, whose length is 10.54 ± 2.08 cm and diameter *D*_u_ is 1.87 ± 0.47 cm. To simulate the living environment, we use the sands dug from the beach in Tangdao Bay, Qingdao, and the sands radius is 0.36 ± 0.14 mm. *U. unicinctus* are 18 cm below the water surface.

### 2.2. Experimental Observation

We use a camera (Canon SX240HS) to record the burrowing behavior of *U. unicinctus* under the sands. Because the sand particle is opaque, it is difficult to observe the burrowing behavior of *U. unicinctus*. Thus, we put *U. unicinctus* in a narrow transparent acrylic box of 200 mm in length, 40 mm in width, and 300 mm in height with sands of 200 mm in height. The narrow box will make it easier for the animal to burrow near the transparent wall for observation. The microscopic images of the skin surface are captured by the extended depth-of-field microscope, LY-WN-YH3D, from Chengdu Li Yang Precision Machinery Co. Ltd.

### 2.3. Uniaxial Tensile Test of the Skin 

Skin samples are cut longitudinally and circumferentially from *U. unicinctus*. The skin samples are clamped by the fixture in the universal testing machine (UTM-1432). The surface of the jaw is serrated with 1.02 mm width and 0.78 mm depth, which can prevent the slipping of the skin. The jaw is closed by rotating the handle on it. The loading velocity is 20 mm min^−1^, and the loading process is kept in a quasistatic state [35]. Removing the clamped length, we denote the initial effective length of the skin by *l*_0_ and the stretched length by *l*. Then, the engineering strain can be given as *ε*= (*l*–*l*_0_)/*l*_0_.

### 2.4. Radial Expansion Pressure Measurement

The balloon is 30.53 ± 0.04 cm in length and 0.61 ± 0.01 cm in diameter. A 50-mL needle tube with an inner diameter of 2.921 ± 0.02 cm is connected to the balloon through a plastic tube, where thin wires are used for water leakage. The balloon is buried under sands at different depths in the acrylic box to simulate the burrowing behavior of *U. unicinctus*. A force gauge (ZP-100 N, with a precision of 0.01 N) is used to measure the highest thrust of the syringe piston during the injection.

### 2.5. Establishment of the FEM–DEM Coupling Model

The software Abaqus is utilized to simulate the burrowing behavior of *U. unicinctus*. For simplification, the sands are viewed as spherical particles simulated by the discrete element PD3D. This kind of element type can be created with specific modifications to the input file [36–40]. We create the part that needs to be discretized, perform mesh division, replace the created node set with point mass/inertia, and change the MASS element type in the generated input file to PD3D. Finally, the discrete element part is obtained. The density of sands is measured as 2.92 ± 0.08 g cm^−3^, and the friction efficiency among sands is 0.25 [41]. *U. unicinctus* skin is simulated by the finite element C3D8R. To obtain accurate results, we use a hyperelastic constitutive relation of the *U. unicinctus* skin in the numerical simulation, which is chosen as the Yeoh model to simulate the large deformation. The initial skin thickness is measured as 1.75 ± 0.19 cm.

## 3. Results and Discussion

### 3.1. Burrowing Behavior and Radial Expansion

It is observed that *U. unicinctus* can expand and shrink by absorbing and spitting water, forming the peristaltic motion. As shown in Figure 1(a), the head of *U. unicinctus* will expand in a radial direction, creating an expansion area of 2 cm in length and 2.5 cm in diameter. Then, the head shrinks and moves forward in the sands, forming a complete peristaltic cycle. The radial expansion and advancement are carried out alternately (Figure 1(b)). *U. unicinctus* can finish one cyclic process within 5 s, advancing about 1 mm each time. The expansion drives the surrounding sands to move radially outward, while the head front face retreats slightly. Although this radial expansion can not directly advance *U. unicinctus* forward, the motion will provide more space for the sands at the front of the head, creating a fluidized area around the animal [42]. One sand particle trajectory, as shown in Figure 1(c), shows that radial expansion will make the squeezed sands separate from each other and start to flow. This phenomenon indicates that the interaction force among the sands weakens, decreasing the pressure *p* of the sands on the head front face. Then, the semicylindrical snout of the head will become thinner, reducing the pressure area *A*. Based on the equation *F* = *pA*, the force *F* for burrowing forward will drop significantly, making it easy to dig into the sands. Finally, *U. unicinctus* repeats the above radial expansion and shrink action to ensure smooth burrowing.

### 3.2. The Fundaments of Radial Expansion

The large deformation of *U. unicinctus* skin provides a basis for their radial expansion in burrowing behavior under the sands. Therefore, it is necessary to study the mechanical properties of skin for further understanding. The uniaxial tensile tests of the skin demonstrate the relationship between Cauchy stress *σ* and the engineering strain *ε*, as shown in Figure 2(a). The skin's longitudinal and circumferential strain values are 3.49 ± 0.16 and 3.61 ± 0.18, respectively. These values are significantly superior to those of reported animals in nature, such as human skin (*ε* = 1.2), rat skin (*ε* = 1.1) [43], and pufferfish skin (*ε* = 0.5) [44]. Only the leech longitudinal skin (*ε* = 3.5) can match these large strain values [45].

Moreover, the stress–strain relation curve shows that the strain increases rapidly and the stress does not change much at the initial stage. Then, the curve slope becomes steeper, and the value roughly becomes a constant. It may be due to the change of polygonal bugles, as shown in Figure 2(a). Initially, polygonal bulges such as pentagons and hexagons are distributed on the skin's surface. These polygonal bulges make the skin highly extensible and stretchable. When the tension starts, the muscles hidden in the polygonal bulges of the skin spread, causing a rapid increase in strain. These polygonal bulges will gradually decrease in height, and they finally disappear with the surface becoming smooth. The skin has already been fully stretched in this phase and begins to endure more stress, so Young's modulus becomes bigger. Meanwhile, the polygonal bugles are randomly distributed on the skin without a specific direction, so the skin is isotropic in terms of macroscopic mechanics. The skin strengths in the longitudinal and circumferential directions are 0.75 ± 0.02 and 0.78 ± 0.02 MPa, which are also similar.

To provide insights into the mechanism of large deformation, we establish the constitutive model of *U. unicinctus* skin. To simplify the analysis, the skin can be viewed as an isotropic material on the macroscale [22, 23]. The skin's mechanical properties are usually associated with the strain energy density *U*. Since the radial expansion is the basis of the *U. unicinctus* burrowing, the tensile experimental data in the circumferential direction are selected to obtain the constitutive model. For incompressible media, the general expression of the strain energy density *U* is given as follows:

(1) $$\begin{array}{c} U=\sum_{i+j=1}^{N}C_{ij}{\left(I_{1}-3\right)}^{i}{\left(I_{2}-3\right)}^{j}, \end{array}$$

where *C*_*ij*_ denotes the material parameter, which can be obtained by fitting the experimental data [46]. The symbols *I*_1_ and *I*_2_ are the first and second invariants of the Cauchy–Green deformation tensor, respectively. They can be expanded in the following form:

(2) $$\begin{array}{c} I_{1}=\lambda_{1}^{2}+\lambda_{2}^{2}+\lambda_{3}^{2}I_{2}=\lambda_{1}^{2}\lambda_{2}^{2}+\lambda_{2}^{2}\lambda_{3}^{2}+\lambda_{3}^{2}\lambda_{1}^{2}, \end{array}$$

where the elongation ratio *λ*_*i*_=1+*ε*_*i*_ (*i* = 1, 2, 3), and *ε*_*i*_ is the principal engineering strain in each principal direction. Meanwhile, the relationship between the Cauhcy stress *σ* and *λ* is given as follows[47, 48]:

(3) $$\begin{array}{c} \sigma =-pI+2\frac{\partial U}{\partial I_{1}}b-2\frac{\partial U}{\partial I_{2}}b^{-1}, \end{array}$$

where $b=\left[\begin{array}{ccc} \lambda_{1}^{2} & 0 & 0\\ 0 & \lambda_{2}^{2} & 0\\ 0 & 0 & \lambda_{3}^{2} \end{array}\right]$and $b^{-1}=\left[\begin{array}{ccc} \lambda_{1}^{-2} & 0 & 0\\ 0 & \lambda_{2}^{-2} & 0\\ 0 & 0 & \lambda_{3}^{-2} \end{array}\right]$. The Formula 3 can also be expressed as follows:

(4) $$\begin{array}{c} \sigma_{i}=-p+2\frac{\partial U}{\partial I_{1}}\lambda_{i}^{2}-2\frac{\partial U}{\partial I_{2}}\lambda_{i}^{-2}, \end{array}$$

where *i* = 1, 2, 3. To eliminate the parameter *p*, the equations with different subscripts will need to be subtracted from each other as follows:

(5) $$\begin{array}{c} \frac{\sigma_{i}-\sigma_{j}}{\lambda_{i}^{2}-\lambda_{j}^{2}}=2\left(\frac{\partial U}{\partial I_{1}}+\lambda_{k}^{2}\frac{\partial U}{\partial I_{2}}\right), \end{array}$$

where *j*, *k* = 1, 2, 3, *λ*_*i*_*λ*_*j*_*λ*_*k*_=1, and *i* ≠ *j* ≠ *k*. Under uniaxial tensile test conditions with tensile direction 1, *λ*_1_^2^=*λ*^2^, *λ*_2_^2^=*λ*_3_^2^=*λ*^−1^, *σ*_2_=*σ*_3_=0, where the first principal elongation ratio *λ*=1+*ε*. *ε* is the first principal engineering strain in the principal direction. The Formula 5 can be simplified as follows:

(6) $$\begin{array}{c} \sigma_{1}=2\left(\lambda^{2}-\lambda^{-1}\right)\left(\frac{\partial U}{\partial I_{1}}+\lambda^{-1}\frac{\partial U}{\partial I_{2}}\right). \end{array}$$

The symbols *I*_1_ and *I*_2_ can be simplified in the following form given as follows:

(7) $$\begin{array}{c} I_{1}=\lambda^{2}+2\lambda^{-1}I_{2}=\lambda^{-2}+2\lambda \;. \end{array}$$

The strain energy density will become the Mooney–Rivlin model *U*_MR_=*C*_10_(*I*_1_ − 3)+*C*_01_(*I*_2_ − 3) when *N* = 1 and *j* = 0, namely:

(8) $$\begin{array}{c} \sigma_{\text{MR}}=2\left(\lambda^{2}-\lambda^{-1}\right)\left(\frac{\partial U_{\text{MR}}}{\partial I_{1}}+\lambda^{-1}\frac{\partial U_{\text{MR}}}{\partial I_{2}}\right)=2\left[{\left(1+\varepsilon \right)}^{2}-{\left(1+\varepsilon \right)}^{-1}\right]\left[C_{10}+C_{01}{\left(1+\varepsilon \right)}^{-1}\right]. \end{array}$$

The strain energy density function also has a reduced polynomial form. When *N* = 1 and *j* = 0, we can obtain the Neo-Hookean model *U*_NH_=*C*_10_(*I*_1_ − 3). The corresponding Cauchy stress can be expressed as follows:

(9) $$\begin{array}{c} \sigma_{\text{NH}}=2\left(\lambda^{2}-\lambda^{-1}\right)\frac{\partial U_{\text{NH}}}{\partial I_{1}}=2C_{10}\left[{\left(1+\varepsilon \right)}^{2}-{\left(1+\varepsilon \right)}^{-1}\right]. \end{array}$$

When *N* = 3 and *j* = 0, we can obtain the Yeoh model *U*_Y_=*C*_10_(*I*_1_ − 3)+*C*_20_(*I*_1_ − 3)^2^+*C*_30_(*I*_1_ − 3)^3^. The corresponding Cauchy stress can be expressed as follows:

(10) $$\begin{array}{c} \sigma_{Y}=2\left(\lambda^{2}-\lambda^{-1}\right)\frac{\partial U_{Y}}{\partial I_{1}}=2\left[{\left(1+\varepsilon \right)}^{2}-{\left(1+\varepsilon \right)}^{-1}\right]\left\{C_{10}+2C_{20}\left[{\left(1+\varepsilon \right)}^{2}+2{\left(1+\varepsilon \right)}^{-1}-3\right]|+3C_{30}{\left[{\left(1+\varepsilon \right)}^{2}+2{\left(1+\varepsilon \right)}^{-1}-3\right]}^{2}\right\}. \end{array}$$

The software Origin is used to fit the uniaxial stress–strain data to obtain the material parameter *C*_*ij*_, as shown in Table 1. The condition for Drucker stability is satisfied by the inequality [49]:

(11) $$\begin{array}{c} \sum_{i=1}^{3}\sum_{j=1}^{3}d\sigma_{ij}d\varepsilon_{ij}>0. \end{array}$$

Under uniaxial tensile test conditions with tensile direction 1, the Formula 11 can be simplified as follows:

(12) $$\begin{array}{c} d\sigma_{1}d\varepsilon_{1}>0. \end{array}$$

This means that the slope of the strain–stress curve needs to be positive. As for the Yeoh model, the slope can be expressed as follows:

(13) $$\begin{array}{c} \frac{d\sigma_{Y}}{d\varepsilon }=\left[2\left(1+\varepsilon \right)+{\left(1+\varepsilon \right)}^{-2}\right]\left\{2\left(C_{10}-6C_{20}+27C_{30}\right)\right.+8\left(C_{20}-9C_{30}\right)\times \left[{\left(1+\varepsilon \right)}^{2}-{\left(1+\varepsilon \right)}^{-1}\right]+18C_{30}\left[{\left(1+\varepsilon \right)}^{2}-{\left(1+\varepsilon \right)}^{-1}\right]. \end{array}$$

As for the Mooney–Rivlin model, the slope can be expressed as follows:

(14) $$\begin{array}{c} \frac{d\sigma_{\text{MR}}}{d\varepsilon }=2\left[2\left(1+\varepsilon \right)+{\left(1+\varepsilon \right)}^{-2}\right]\times \left[C_{10}+C_{01}{\left(1+\varepsilon \right)}^{-1}\right]-2C_{01}\left[{\left(1+\varepsilon \right)}^{2}-{\left(1+\varepsilon \right)}^{-1}\right]\times {\left(1+\varepsilon \right)}^{-2} \end{array}$$

As for the Neo-Hookean model, the slope can be expressed as follows:

(15) $$\begin{array}{c} \frac{d\sigma_{\text{NH}}}{d\varepsilon }=2C_{10}\left[2\left(1+\varepsilon \right)+{\left(1+\varepsilon \right)}^{-2}\right]. \end{array}$$

Based on the data, as shown in Table 1, the slopes of the Neo-Hookean model and the Yeoh model are always positive while the slope of the Mooney–Rivlin model is sometimes negative. This means that the Neo-Hookean model and the Yeoh model are stable, while the Mooney–Rivlin model is unstable. In the case of negative *C*_20_, the Yeoh model is also applicable if *U* increases monotonically with the deformation [24, 49, 50]. These fitting curves are shown in Figure 2(b), implying that the Yeoh model is closest to the experimental data. Thus, the constitutive model of skin can be expressed as follows:

(16) $$\begin{array}{c} \sigma_{Y}=2\left[{\left(1+\varepsilon \right)}^{2}-{\left(1+\varepsilon \right)}^{-1}\right]\left\{8.84\times 10^{-3}-6.28\times 10^{-4}\times |\left[{\left(1+\varepsilon \right)}^{2}|+2{\left(1+\varepsilon \right)}^{-1}-3\right]+7.11\times 10^{-5}\times \left[{\left(1+\varepsilon \right)}^{2}+2{\left(1+\varepsilon \right)}^{-1}-3\right]\right\}. \end{array}$$

In addition to the skin's large deformation, *U. unicinctus* needs to apply enough pressure to surrounding sands to radially expand so that they can move forward continuously. However, it is hard to measure this pressure directly. Thus, similar expansion experiments are performed with a latex balloon (purchased from Tmall) instead of *U. unicinctus* to explore the relationship between burrowing depth and expansion pressure. To simulate the water absorption process of *U. unicinctus*, we slowly inject water into the balloon, increasing the inner pressure and inflating the balloon near the plastic tube, as shown in Figure 2(c). The final injection volume of water is 9.8 mL to form an expansion zone similar in volume to *U. unicinctus*, making the surrounding sands move radially outward. The forces *F*_p_ under the sands at the depth *h* = 0, 4, 5, 7, and 10 cm are 9.10 ± 0.48, 11.69 ± 0.83, 12.57 ± 1.08, 13.95 ± 0.70, and 15.18 ± 1.62 N. Since the syringe piston area *A*_p_ = *πD*_*p*_^2^/4 = 6.70 cm^2^, the internal pressures in the balloon at different depths can be obtained by dividing the force *F*_p_ by the area *A*_p_, which are 13.59 ± 0.71, 17.45 ± 1.24, 18.77 ± 1.61, 20.83 ± 1.05, and 22.66 ± 2.42 kPa, respectively. The internal pressure at the depth *h* = 0 cm is induced by the expansion of the balloon itself. Therefore, the actual external pressures *p*_e_ for the radial expansion at the depth *h* = 4, 5, 7, and 10 cm are 11.69 ± 1.24, 12.57 ± 1.61, 13.95 ± 1.05, and 15.18 ± 2.42 kPa, respectively. Therefore, as the depth increases, the expansion pressure of *U. unicinctus* will increase linearly. The relationship between the external pressure *p*_e_ and the depth *h* can be expressed as *p*_*e*_ *=* kh, where *k* = 0.97 kPa cm^−1^.

### 3.3. The Effect of Radial Expansion on Burrowing: FEM–DEM Coupling Simulation

Based on the constitutive model of *U. unicinctus* skin, we utilize the software Abaqus to obtain the expansion pressure to uncover the mechanism of burrowing. We establish the finite element method–discrete element method (FEM–DEM) coupling model of burrowing and get the von Mises stress cloud diagram under the 4 cm depth sands, as shown in Figure 3(a). The white particles represent the sands, and the blue zone represents *U. unicinctus* skin. The skin will expand from 1.87 to 2.5 cm in diameter *D*_u_. An expansion area is formed at 18 cm underwater, whose length is 2 cm. As the diameter *D*_u_ increases, the stress in the skin will increase, where greater stress is concentrated in the more curved areas of the skin. When *U. unicinctus* expands to its maximum size, the skin's maximum stress, 0.042 MPa, is an order of magnitude smaller than the skin's strength, implying that the skin is strong enough in the burrowing process.

The internal and external pressures on the *U. unicinctus* skin under the 4 cm depth sands are shown in Figure 3(b). Interestingly, we can see that the external pressure does not always increase with the radial expansion. Initially, the interaction among the particles is relatively strong, so the external pressure *p*_e_ will increase linearly with the increase in the diameter *D*_u_, as shown by the solid blue line in Figure 3(b). Then, the surrounding particles will gradually move relative to each other, and the forces among them will gradually decrease, making the slope of the curve decrease progressively. Finally, when all surrounding particles are misaligned and moved, the pressure curvature will no longer increase. Similarly, the internal pressure *p*_i_ also increases linearly at the beginning. There is a slight difference between the internal and external pressures due to the small Young's modulus of the *U. unicinctus* skin at the initial stage, as shown by the red dash line in Figure 3(b). Subsequently, the internal pressure will increase with a lower growth rate. At this stage, the Young's modulus of the skin of *U. unicinctus* becomes large. The increasing skin strain contributes to the growing gap between the internal and external pressures. At the final stage, the internal pressure can reach 4.06 kPa. In addition to the simulation example at 4 cm depth, we also simulate the expansion process at 5, 7, and 10 cm depth. As shown in Figure 3(c), the simulated external pressure curve is very similar to the experimental curve, verifying the correctness of the simulation.

The purpose of the radial expansion is to move forward under sands. The displacement cloud diagram under the 4 cm depth sands is shown in Figure 4(a). As the diameter increases, the head of *U. unicinctus* will recede so that the sands will collapse and follow to move right, as shown in the red area. The displacement vector, as shown in Figure 4(b), indicates the fluidized zone of the sands more clearly, where the trajectory of sands is similar to the experimental phenomenon, as shown in Figure 2(c). The relationship between the head receding distance *D*_r_ and the diameter *D*_u_ is represented by the solid blue line, as shown in Figure 5. Interestingly, as the diameter increases, the initial receding distance of the head is relatively small. This phenomenon may be since the initial pull force on the head is small, considering the constitutive relationship of the skin. As *U. unicinctus* expands radially, the pressure of sand particles on the head *p*_h_ will drop rapidly by 97.7% at the initial stage and remain stable when the diameter exceeds about 2.2 cm, represented by the red dash line in Figure 5. It is worth mentioning that the pressure drop on the head is mainly at the stage of the sand particles from rest to collapse. After that, the pressure stabilizes instead. The radial expansion will reduce the pressures at the depth *h* = 5, 7, and 10 cm by 96.8%, 96.4%, and 97.4%, respectively, and the resistance pressure is only 25 ± 8.5 Pa when *U. unicinctus* start to move forward.

## 4. Conclusion

*U. unicinctus* can burrow U-shaped channels on the seabed for predation and defense. In this process, *U. unicinctus* utilizes the skin's large deformation to expand radially, causing the sands to collapse and reducing the pressure on the head. This behavior will make it easy to move forward in the fluidized area of the sands. Uniaxial tensile tests show that the skin strain can reach about 3.5 due to the excess skin stored in the bulges. The stress–strain relationship can be expressed by the Yeoh model, with *R*^2^ = 0.995. Considering the large deformation of the skin and the discrete nature of the sands, we establish the FEM–DEM coupling model based on Abaqus software to study the effect of radial expansion on the burrowing behavior. The results show that the simulated external pressure for radial expansion increases with the burrowing depth and is very close to the experimental pressure, implying the reliability of the simulation. What surprised us is that the radial expansion can drastically reduce the pressure of sand particles on the head front face to about 1/35 of the initial value. Considering that the head surface area will shrink when moving forward, the radial expansion will significantly decrease the difficulty of burrowing. This burrow method of *U. unicinctus* can pave a new way for engineering burrowing devices and intelligent robots in loose foundations.

## Figures and Tables

**Figure 1:** The burrowing behavior of *Urechis unicinctu*s under the sand. (a) *Urechis unicinctu*s can advance in sands by peristaltic motion. (b) The radial expansion and the advancement of the head are carried out alternately. (c) The trajectory of one sand particle near the head shows that the radial expansion can make the sands flow.

**Figure 2:** The large deformation of *Urechis unicinctus* skin. (a) The polygonal structure on the skin surface is the basis for the skin's large deformation, and the longitudinal stress–strain relationship of the skin is similar to the circular. (b) Among the stress–strain fitting curves of the skin, the Yeoh model fits with the experimental data best. (c) Balloon expansion tests under the sands are used to indirectly measure the pressure required for the radial expansion of *Urechis unicinctu*s.

**Figure 3:** The stress simulation result. (a) The radial movement of *Urechis unicinctus* places greater stress on the skin near the expansion area, especially for the sections with high curvature. (b) The internal and external pressures on the skin increase with the radial movement under the 4 cm depth sand, but the rate of increase decreases gradually. (c) As for the relationship between external pressure and drilling depth, the simulation results are very close to the experimental results, proving the reliability of the simulation.

**Figure 4:** The displacement simulation result. (a) The radial expansion collapses surrounding sands and makes them move, especially for the sands near the head front face. The local displacement field of the sands in (b) clearly shows the trajectory of these particles.

**Figure 5:** The influence of the expansion distance on the head front pressure and the head receding distance. The pressure drop is mainly located at the initial stage of the radial expansion, but the head receding distance is small at this stage.

**Table 1:** The material parameters in constitutive models indicate that the Yeoh model is best suited for the skin constitutive model.

The material parameter	*C*_01_ × 10^−4^	*C*_10_ × 10^−4^	*C*_20_ × 10^−4^	*C*_30_ × 10^−4^	*R* ^2^	Stability
The Mooney–Rivlin model	−585 ± 94.20	293 ± 25.50			0.911	Unstable
The Neo-Hookean model		138 ± 7.78			0.815	Stable
The Yeoh model		88.4 ± 8.06	−3.19 ± 0.75	0.24 ± 0.02	0.995	Stable

## Data Availability

All data included in this study are available upon request by contact with the corresponding authors.
